# GLP2 Promotes Directed Differentiation from Osteosarcoma Cells to Osteoblasts and Inhibits Growth of Osteosarcoma Cells

This article has been retracted.

**DOI:** 10.1016/j.omtn.2017.12.009

**Published:** 2017-12-21

**Authors:** Yi Lu, Dongdong Lu, Yu Hu

**Affiliations:** 1 Department of Geriatrics, Zhongshan Hospital, Fudan University, Shanghai 200032, China; 2 School of Life Science and Technology, Tongji University, Shanghai 200092, China

**Keywords:** glucagon-like peptide 2, osteosarcoma, osteoblast, c-Fos, BMP, NF-κB

## Abstract

Glucagon-like peptide 2 (GLP2) is a proglucagon-derived peptide that is involved in the regulation of energy absorption and exerts beneficial effects on glucose metabolism. However, the exact mechanisms underlying the GLP2 during osteogenic differentiation has not been illustrated. Herein, we indicated that GLP2 was demonstrated to result in positive action during the osteogenic differentiation of human osteosarcoma cells. Our findings demonstrate that GLP2 inhibis the growth of osteosarcoma cells *in vivo* and *in vitro*. Mechanistic investigations reveal GLP2 inhibits the expression and activity of nuclear factor κB (NF-κB), triggering the decrease of c-Myc, PKM2, and CyclinD1 in osteosarcoma cells. In particular, rescued NF-κB abrogates the functions of GLP2 in osteosarcoma cells. Strikingly, GLP2 overexpression significantly increased the expression of osteogenesis-associated genes (e.g., Ocn and PICP) dependent on c-Fos-BMP signaling, which promotes directed differentiation from osteosarcoma cells to osteoblasts with higher alkaline phosphatase activity. Taken together, our results suggested that GLP2 could be a valuable drug to promote directed differentiation from osteosarcoma cells to osteoblasts, which may provide potential therapeutic targets for the treatment of osteosarcoma.

## Introduction

Osteoblasts (OBs) are specialized, terminally differentiated products of mesenchymal stem cells.^1^ It is an important store of minerals for physiological homeostasis, including both acid-base balance and calcium or phosphate maintenance.^2^, ^3^ A study showed that osteochondroprogenitor cells could differentiate under the influence of growth factors, e.g., Cbfa1/Runx2. Moreover, key growth factors, e.g., bone morphogenetic proteins (BMPs) and sclerostin, were involved in skeletal differentiation.^4^ Furthermore, studies indicate osteosarcomas tend to occur at the sites of bone growth, presumably because proliferation makes osteoblastic cells in this region.^5^ Strikingly, multipotent adult progenitor cells on an allograft scaffold may facilitate the bone repair process.^6^ In addition, osteogenic differentiation of human mesenchymal stem cells promotes mineralization within a biodegradable peptide hydrogel.^7^ Strikingly, miR-34a promotes osteogenic differentiation of human adipose-derived stem cells via the RBP2/NOTCH1/CyclinD1 coregulatory network,^8^ and Pioglitazone (PIO) (a thiazolidinedione) may also promote osteoclastogenesis by affecting the osteoprotegerin (OPG)/receptor activator of nuclear factor κB ligand (RANKL)/RANK (OPG-RANKL-RANK) system.^9^

GLP2, a glucagon (GCG) peptide family member, is related to the regulation of energy absorption and maintenance of mucosal morphology and functions. Indeed, GLP2 acts as a beneficial factor for glucose metabolism in mice with high-fat diet-induced obesity.^10^ Moreover, GLP2 exhibits a protective effect on hepatic ischemia-reperfusion injury in rats,^11^ and GLP2 agonists decrease the need for parenteral nutrition (PN) in short bowel syndrome (SBS).^12^, ^13^ Furthermore, the absence of a motif in GLP2 could be the reason for a significantly lower strength of interaction between GLP2 and heparin in inducing protein aggregation.^14^ In particular, alteration of the intestinal barrier and GLP2 secretion was found in Berberine-treated type 2 diabetic rats.^15^ Notably, GLP2-2G-XTEN is efficacy in a rat Crohn’s disease model requiring a lower molar dose and less frequent dosing relative to GLP2-2G peptide.^16^ Interestingly, endogenous GLP2 is a key mediator of refeeding-induced and resection-induced intestinal adaptive growth.^17^ Intriguingly, GLP2 elicits neuroprotective effects on rat myenteric neurons cultured with or without mast cells by activating separate receptors VIP.^18^ On the other hand, the evidence that suppressor of cytokine-signaling protein is induced by GLP2 in normal or inflamed intestine may limit IGF1-induced growth but protect against risk of dysplasia or fibrosis.^19^ Significantly, studies also showed GLP2 could reduce food intake in mice in the short term, likely acting at a peripheral level.^20^

At the present, the exact mechanisms underlying the GLP2 during osteogenic differentiation are not fully illustrated. The aim of this study was to explore the role of GLP2 in the control of OB differenitiation and to validate how this molecule could exert protective effects against the onset of osteosarcoma.

## Results

### GLP2 Inhibits Osteosarcoma Cell Growth *In Vivo* and *In Vitro*

To address whether the GLP2 impacts on malignant proliferation of osteosarcoma cells, we prepared the rLV-GLP2 lentivirus (Figure 1A), and we established the stable osteosarcoma cell line (MG63) infected with rLV or rLV-GLP2, respectively (Figure 1B). GLP2 was significantly overexpressed in MG63 infected with rLV-GLP2 compared to the control (Figure 1C). Using ELISA, we measured GLP2 released by the MG63 cells before and after transduction of GLP2. The results showed that the released level of GLP2 in the rLV-GLP2-infected group was significantly higher than in the rLV control group (0 versus 696.78 ± 152.77 pg/mL; p = 0.0078244 < 0.01) (Figure S1A). Furthermore, GLP2R was expressed in MG63 cells, and there was no significant difference between the rLV group and the rLV-GLP2 group (Figure S1B). Moreover, the interaction between GLP2 and GLP2R was significantly detected in MG63 cells infected with rLV-GLP2, but not in MG63 cells infected with rLV (Figure 1D). At the first time, we detected these cells’ proliferation ability *in vitro*. As shown in Figure 1E, overexpression of GLP2 significantly decreased proliferation ability of MG63 (p < 0.01). The BrdU staining findings showed that the BrdU-positive rate was 18.87% ± 5.75% in the rLV-GLP2 group, and the BrdU-positive rate was 49.4% ± 9.73% in the control rLV group (p < 0.01) (Figure 1F). Then we conducted soft agar colony formation efficiency assay in these cells. The soft agar colony formation rate was 20.63% ± 3.06% in GLP2-overexpressed MG63 cells; in contrast, the soft agar colony formation rate was 60.77% ± 6.07% in the control rLV group (p = 0.0069 < 0.01) (Figure 1G). Furthermore, the cell transwell rate was 7.2% ± 1.55% in the rLV GLP2 group, and the cell transwell rate was 23.08% ± 5.43% in the control rLV group (p < 0.01) (Figure 1H).

**Figure 1:** GLP2 Inhibits Osteosarcoma Carcinogenesis *In Vitro* (A) The photography of the HEK293 cell lines infected with rLV-Green-GLP2. (B) The photography of the MG63 cell lines infected with rLV-Green or rLV-Green-GLP2. (C) Western blotting with anti-GLP2 in MG63 infected with rLV-GLP2 or rLV. β-actin was used as an internal control. (D) Co-Immunoprecipitation (coIP) with anti-GLP2R followed by western blotting with anti-GLP2 in MG63 cells infected with rLV or rLV-GLP2. IgG IP as negative control. INPUT refers to western blotting with anti-GLP2 and anti-GLP2R. (E) Cell proliferation assay was performed in 96-well format using the CCK8 cells proliferation kit to determine the cell viability as described by the manufacturer. Each sample was assayed in triplicates for 3 days consecutively.Cell growth curve was based on the corresponding the relative values of OD450 and each point represents the mean of three independent samples. Data are means of value from three independent experiments (error bar ± SEM; *p < 0.05). (F) Cell BrdU assay. Data are means of value from three independent experiment (error bar ± SEM; **p < 0.01). (G) (left)The photography of colonies from the cell lines indicated in left. (right) Cell plate colony formation ability assay. Data are means of value from three independent experiment, bar ± SEM. (H) Cell transwell assay. Data are means of value from three independent experiment (error bar ± SEM; **p < 0.01).

To further validate the effect of GLP2 on osteosarcoma carcinogenesis *in vivo*, the stable MG63 cells lines with altered expression of GLP2 were injected subcutaneously into athymic BALB/c nude mice. As shown in Figure 2A, when GLP2 was overexpressed, the xenograft tumor weight decreased approximately 5-fold compared to the corresponding control group (0.15 ± 0.04 g versus 0.73 ± 0.14 g; p < 0.01). Compared to the control group, excessive GLP2 increased the time of xenograft tumor formation (14.5 ± 3.05 days versus 9.22 ± 1.59 days; p < 0.01) (Figure 2B). Moreover, xenograft tumor had more well differentiation cells in the GLP2-overexpressing group than that of the control group. The proliferation index (calculated as a percentage of PCNA-positive cells) was significantly lower in GLP2-overexpressing xenograft tumors compared to the control rLV group (20% ± 3.92% versus 53.59% ± 10.28%; p < 0.01) (Figure 2C). In particular, our results also showed that excessive GLP2 inhibited the growth of orthotopic osteosarcoma. when GLP2 was overexpressed, the weight of orthotopic osteosarcoma decreased approximately 3-fold when compared to the corresponding control group (0.586 ± 0.137 g versus 0.192 ± 0.06 g; p = 0.000002 < 0.01) (Figure S2A), and the tumor formation time of the rLV group (7.2 ± 1.39 days) was shorter than that of the rLV-GLP2 group (13 ± 2.67 days; p = 0.00008 < 0.01) (Figure S2B). Together, these findings suggest that GLP2 inhibits growth of osteosarcoma cells *in vivo* and *in vitro*.

**Figure 2:** GLP2 Inhibits Osteosarcoma Carcinogenesis *In Vivo* (A) The xenograft tumors from BALB/c mouse injected with MG63 cells infected with rLV-GLP2 or rLV. subcutaneously at armpit. The xenograft tumors weight (gram) in the two groups. Data were means of value from ten BALB/c mice (mean ± SEM; n = 10; **p < 0.01). (B) The xenograft tumors appearance time in the two groups. Data were means of value from ten BALB/c mice (mean ± SEM; n = 10; *p < 0.05). (C) A portion of each xenograft tumor was fixed in 4% formaldehyde and embedded in paraffin, and the micrometers of sections (4 μm) were made for PCNA staining (original magnification × 100). **p < 0.01.

### GLP2 Inhibits the Expression of NF-κB in Osteosarcoma Cells

Given that GLP2 inhibited malignant growth of osteosarcoma cells, we considered whether this function is associated with inflammation-related genes, e.g., nuclear factor κB (NF-κB). In the cell lines, GLP2 was significantly overexpressed in MG63 infected with rLV-GLP2 compared to the control MG63 infected with rLV (Figure S3). As shown in Figure 3A, the excessive GLP2 significantly inhibited the loading of RNA polymerase II (Pol II) onto the NF-κB promoter region compared to the control group. Moreover, the excessive expression of GLP2 significantly decreased the luciferase activity of NF-κB promoter compared to control (Figure 3B). Furthermore, we performed western blotting and RT-PCR assay; the excessive expression of GLP2 significantly reduced the level of transcription and translation of NF-κB compared to control (Figure 3C). Significantly, through co-immunoprecipitation (coIP) with anti-NF-κB, the excessive expression of GLP2 significantly decreased the binding of NF-κB to β-catenin or AP1 compared to control (Figure 3D). Furthermore, through chromatin immunoprecipitation (ChIP) assay with anti-NF-κB, the excessive expression of GLP2 significantly decreased the loading of NF-κB onto the promoter region of c-Myc, PKM2, and CyclinD1 compared to control (Figure 3E). Ultimately, the excessive GLP2 significantly decreased the level of transcription and translation of c-Myc, PKM2, and CyclinD1 compared to control (Figures 3F and 3G). Taken together, these observations suggest that GLP2 inhibits the expression and activity of NF-κB in osteosarcoma cells.

**Figure 3:** GLP2 Inhibits the Expression of NF-κB in MG63 (A) ChIP assay with anti-RNA polII followed by PCR with promoter DNA primers of NF-κB in MG63 cells infected with rLV-GLP2 or rLV. IgG ChIP was the negative control. NF-κB promoter as INPUT. (B) The assay of luciferase activity of prmoter of NF-κB in MG63 infected with rLV-GLP2 or rLV, respectively. Data are means of value from three independent experiment (error bar ± SEM; **p < 0.01). (C) Western blotting with anti-NF-κB and RT-PCR with NF-κB primers in MG63 infected with rLV-GLP2 or rLV. β-actin as internal control. (D) Co-immunoprecipitation (coIP) with anti-NF-κB followed by western blotting with anti-β-catenin and anti-AP1 in MG63 infected with rLV-GLP2 or rLV, respectively. IgG IP was used as a negative control. INPUT refers to western blotting with anti-β-catenin and anti-AP1. (E) ChIP assay with anti-NF-κB followed by PCR with DNA primers (promoter region) of c-Myc,PKM2, CyclinD1 in MG63 cells infected with rLV-GLP2 or rLV. IgG ChIP was the negative control. The promoters of c-Myc, PKM2, CyclinD1 as INPUT. (F) RT-PCR with primers of c-Myc, PKM2, CyclinD1 in MG63 infected with rLV-GLP2 or rLV. β-actin as internal control. (G) Western blotting with anti-c-Myc, anti-PKM2, anti-CyclinD1 in MG63 infected with rLV-GLP2 or rLV. β-actin as internal control.

### Excessive NF-κB Abrogates the Function of GLP2 in Osteosarcoma Cells

To validate whether NF-κB blocked the function of GLP2 in osteosarcoma cells, we established the stable MG63 (osteosarcoma cells) infected with rLV, rLV-GLP2, or rLV-GLP2 plus pcDNA3-NF-κB. Using ELISA, we measured GLP2 released by the MG63 cells after co-NF-κB transduction. The results showed that the released level of GLP2 in the rLV-GLP2-infected group was significantly higher than in the control rLV-infected group (0 versus 950.04 ± 62.67 pg/mL; p = 0.0007 < 0.01); however, the released level of GLP2 in the rLV-GLP2-infected group was not significantly altered compared to the rLV-GLP2 plus pcDNA3-NF-κB group (877.13 ± 106.36 versus 950.04 ± 62.67 pg/mL; p = 0.145 > 0.05) (Figure S4A). Furthermore, GLP2R was expressed in MG63 cells, and there was no significant difference among the rLV, rLV-GLP2, and rLV-GLP2 plus pcDNA3-NF-κB groups (Figure S4B). As shown in Figure 4A, compared to the control group, GLP2 was significantly overexpressed in MG63 transfected with rLV-GLP2 and pLV-GLP2 plus pcDNA3-NF-κB, respectively, and NF-κB was significantly decreased in MG63 transfected with rLV-GLP2 and was increased in MG63 infected with pLV-GLP2 plus pcDNA3-NF-κB. At the first time, we detected these cells proliferation ability *in vitro*. As shown in Figure 4B, excessive GLP2 significantly decreased proliferation ability of MG63 (p < 0.01). However, proliferation ability of MG63 was not significantly different between the rLV group and the pLV-GLP2 plus pcDNA3-NF-κB group (p > 0.05). Furthermore, the BrdU staining findings showed that the BrdU-positive rate was 16.06% ± 2.06% in the GLP2-overexpressing group, and the BrdU-positive rate was 57.13% ± 12.73% in the rLV control group (p < 0.01). However, the BrdU-positive rate was 50% ± 5.96% in the pLV-GLP2 plus pcDNA3-NF-κB group (57.13% ± 12.73% versus 50% ± 5.96%; p > 0.05) (Figure 4C). Then we conducted soft agar colony formation efficiency assay in these cells. The soft agar colony formation rate was 21.29% ± 4.07% in the rLV-GLP2 group, and the soft agar colony formation rate was 55.83% ± 12.9% in the rLV group l (p < 0.01). However, the soft agar colony formation rate was 56.19% ± 7.77% in the rLV-GLP2 plus pcDNA3-NF-κB group (55.83% ± 12.9% versus 56.19% ± 7.77%; p > 0.05) (Figure 4D).

**Figure 4:** Excessive NF-κB Abrogates the Function of GLP2 in MG63 *In Vitro* and *In Vivo* (A) Western blotting with anti-GLP2, NF-κB in MG63 infected with rLV-GLP2, rLV-GLP2 plus pcDNA3-NF-κB or pLV. β-actin was used as an internal control. (B) Cell proliferation assay was performed in 96-well format using the CCK8 cells proliferation kit to determine the cell viability as described by the manufacturer. Each sample was assayed in triplicates for 3 days consecutively. Cell growth curve was based on the corresponding the relative values of OD450 and each point represents the mean of three independent samples. Data are means of value from three independent experiments (error bar ± SEM; **p < 0.01 and *p < 0.05). (C) Cell BrdU assay. Data are means of value from three independent experiment (error bar ± SEM; **p < 0.01). (D) Cell plate colony formation ability assay. Data are means of value from three independent experiment (error bar ± SEM; **p < 0.01). (E) The xenograft tumors from BALB/c nude mouse injected with MG63 cells infected with rLV, rLV-GLP2, rLV-GLP2 plus pcDNA3-NF-κB subcutaneously at armpit. The xenograft tumors weight (gram) in the three groups. Data were means of value from six BALB/c mice (mean ± SEM; n = 6; **p < 0.01). (F) A portion of each xenograft tumor was fixed in 4% formaldehyde and embedded in paraffin, and the micrometers of sections (4 μm) were made for PCNA staining (original magnification × 100). **p < 0.01.

Next, the xenograft tumors from BALB/c nude mouse were injected with MG63 cells infected with rLV-GLP2, rLV-GLP2 plus pcDNA3-NF-κB, or rLV subcutaneously at the armpit. As shown in Figure 4E, when GLP2 was overexpressed, the xenograft tumor weight decreased approximately 7-fold compared to the control group (0.125 ± 0.033 g versus 0.833 ± 0.100 g; p < 0.01). However, compared to the control group, xenograft tumor weight was not significantly altered in the rLV-GLP2 plus pcDNA3-NF-κB group (0.79 ± 0.165 g versus 0.833 ± 0.100 g; p > 0.05). Moreover, the PCNA-positive rate of cells was significantly lower in GLP2 overexpressed tumors compared to the control rLV group (25.53% ± 4.38% versus 58.3% ± 10.58%; p < 0.01). However, compared to the control group, PCNA-positive rate was not significantly altered in the rLV-GLP2 plus pcDNA3-NF-κB group (54.63% ± 7.62% versus 58.3% ± 10.58%; p > 0.05) (Figure 4F). Together, these observations demonstrate that excessive NF-κB abrogates the function of GLP2, and the cancerous suppression of GLP2 is regulated and controlled by NF-κB in osteosarcoma cells.

### GLP2 Promotes Directed Differentiation from Osteosarcoma Cells to OBs

To explore whether GLP2 promotes the differentiation of MG63 to OB, we constructed a model of OB induced from the MG63 infected with rLV or rLV-GLP2 using dexamethasone, β-glycerophosphate, and mlascorbic acid (Asc) for 21 days, according to the schematic digram (Figure 5A). Our result showed that GLP2 was significantly overexpressed in OB induced from MG63 infected with rLV-GLP2 compared to the control OB induced from MG63 infected with rLV (Figure 5B). Using ELISA, we measured GLP2 released by the OB cells before and after transduction of GLP2. The results showed that the released level of GLP2 in the rLV-GLP2-infected group was significantly higher than in the rLV-green control group (0 versus 480.53 ± 107.59322 pg/mL; p = 0.0082 < 0.01) (Figure S5A). Furthermore, GLP2R was expressed in OB cells, and there was no significant difference between the rLV group and the rLV-GLP2 group (Figure S5B). Moreover, compared to control, the induced OB cells (bone alkaline phosphatase [BALP]-positive cells) were increased in the rLV-GLP2 group (11.14% ± 2.55% versus 78.23% ± 8.26%; p < 0.01) (Figure 5C). Furthermore, compared to control, the calcific nodules were significantly increased in the rLV-GLP2 group (4.72% ± 1.204% versus 18.19% ± 2.636%; p < 0.01) (Figure 5D). Moreover, compared to control, the transcriptional level of BALP, Ocn, and PICP was significantly increased in the rLV-GLP2 group (Figure 5E), and the expression of BALP, Ocn, and PICP was significantly increased in the rLV-GLP2 group (Figure 5F). Furthermore, the BALP activity was significantly increased in the rLV-GLP2 group (Figure 5G), and the PICP activity was significantly increased in the rLV-GLP2 group (Figure 5H). Taken together, these observations suggest that GLP2 could promote the directed differentiation from osteosarcoma cells to osteoblasts.

**Figure 5:** GLP2 Promotes the Directed Differentiation from MG63 to Osteoblast (OB) (A) The schematic digram illustrates a model of osteoblast induced from human osteosarcoma cell line MG63 with dexamethasone,β- glycerophosphate and mlascorbic acid(Asc) for 21days. (B) Western blotting with anti-GLP2 in induced OB. β-actin as internal control. (C, left) The photography of BALP staining. (C, right). The BALP positive rate. (D, left) The photography of calcific nodules after induction of OB. (D, right) The rate of calcific nodules in OB. (E) RT-PCR analysis for BALP, Ocn and PICP in induced OB.β-actin as internal control. (F) Western blotting with anti-BALP, anti-Ocn, anti-PICP in induced OB. β-actin was used as an internal control. (G) Cell BALP activity assay. Data are means of value from three independent experiment (error bar ± SEM; **p < 0.01). (H) Cell PICP activity assay. Data are means of value from three independent experiment (error bar ± SEM; **p < 0.01).

### GLP2 Enhances the Expression of BMP through c-Fos in OBs

Given that GLP2 could enhance the directed differentiation from osteosarcoma cells to OBs, we tried to validate the involvement of c-Fos and BMP during this differentiation. In the cell lines, GLP2 was significantly overexpressed in OB induced from MG63 infected with rLV-GLP2 compared to the control OB induced from MG63 infected with rLV (Figure S6A). At the first time, we adopted RNA immunoprecipitation (RIP) with anti-METTL3 followed by RT-PCR with FOS primers in OB cells. The results showed that the excessive expression of GLP2 enhanced the binding of METTL3(a mRNAmethyltransferase) to c-Fos mRNA compared to control (Figure 6A). Moreover, we performed RIP with anti-m6A followed by RT-PCR with c-Fos primers in OB cells. The results showed that the excessive expression of GLP2 promoted methylation of the c-Fos mRNA compared to rLV control (Figure 6B). Furthermore, we performed RT-PCR analysis of c-Fos in OB cells, and the results showed that overexpression of GLP2 enhanced the transcription of c-Fos in OB cells compared to control (Figure 6C). Next, we performed western blotting with anti-Fos in OB cells, and the results showed that overexpression of GLP2 enhanced the expression of c-Fos in OB cells compared to control group (Figure 6D). Furthermore, compared to control, excessive GLP2 increased the loading of c-Fos on the promoter region of BMP (Figure 6E). Moreover, compared to control, excessive GLP2 increased the luciferase activity of the promoter of BMP (Figure 6F). Ultimately, compared to control, excessive GLP2 increased the transcription and translation of BMP (Figure 6G).Taken together, GLP2 enhanced the expression of BMP dependent on c-Fos in OB cells.

**Figure 6:** GLP2 Promotes the Expression of BMP Dependent on c-Fos (A) RNA immunoprecipitation (RIP) with anti-METTL3 followed by RT-PCR with c-Fos primers in OB cells induced from MG63 infected with rLV-GLP2 or rLV, respectively. IgG RIP as negative control. RT-PCR for c-Fos as INPUT. (B) RNA Immunoprecipitation(RIP) with anti-m6A followed by RT-PCR with c-Fos primers in OB cells induced from MG63 infected with rLV-GLP2 or rLV, respectively. IgG RIP as negative control. RT-PCR for c-Fos as INPUT. (C) RT-PCR analysis of Fos in OB cells induced from MG63 infected with rLV-GLP2 or rLV, respectively. β-actin as internal control. (D) Western blotting with anti-FOS in OB cells induced from MG63 infected with rLV-GLP2 or rLV, respectively. β-actin was used as an internal control. (E) ChIP assay with anti-FOS followed by PCR with DNA primers of BMP in OB cells induced from MG63 infected with rLV-GLP2 or rLV, respectively. IgG ChIP was the negative control. (F) The assay of luciferase activity of promoter of BMP in OB induced from MG63 infected with rLV-GLP2 or rLV, respectively. **p < 0.01. (G) Western blotting with anti-BMP and RT-PCR with BMP cDNA primers in OB cells induced from MG63 infected with rLV-GLP2 or rLV, respectively. β-actin as internal control.

### GLP2 Activates the BALP and PICP through c-Fos and BMP in OBs

To validate whether GLP2 could alter the transcriptional activity of BALP and PICP, we performed related detection in OBs. In the cell lines, GLP2 was significantly overexpressed in OB induced from MG63 infected with rLV-GLP2 compared to the control OB induced from MG63 infected with rLV (Figure S6B). At the first time, we adopted ChIP assay with anti-c-Fos and anti-BMP followed by PCR with BALP and PICP promoter primers in OB cells induced from MG63 infected with rLV-GLP2 or control OB induced from MG63 infected with rLV, respectively. The results showed that excessive GLP2 increased the loading of FOS or BMP on the promoter region of BALP and PICP compared to the control group (Figure 7A). Furthermore, compared to control, excessive GLP2 increased the luciferase activity of the promoter of BALP (Figure 7B), and excessive GLP2 increased the luciferase activity of the promoter of PICP (Figure 7C). Taken together, these observations suggest that GLP2 enhanced the transcriptional activity of BALP and PICP in OB cells.

**Figure 7:** GLP2 Enhances the Expression of BALP, PICP via c-Fos and BMP (A) ChIP assay with anti-BMP, anti-FOS followed by PCR with DNA primers of BALP and PICP in OB cells induced from MG63 infected with rLV-GLP2 or rLV, respectively. IgG ChIP was the negative control. (B) The assay of luciferase activity of promoter of BALP in OB cells induced from MG63 infected with rLV-GLP2 or rLV, respectively. **p < 0.01. (C) The assay of luciferase activity of promoter of PICP in OB cells induced from MG63 infected with rLV-GLP2 or rLV, respectively. **p < 0.01.

### c-Fos Knockdown Abrogates GLP2 Action in OBs

To validate whether function of GLP2 in OB is elicited by c-Fos, we obtained three stable OB cells induced from MG63 infected with rLV, rLV-GLP2, and rLV-GLP2 plus pGFP-V-RS-c-Fos, respectively. Using ELISA, we measured GLP2 released by the OB cells after c-Fos knockdown. The results showed that the released level of GLP2 in the rLV-GLP2-infected group was significantly higher than in the rLV control group (0 versus 541.01 ± 84.28 pg/mL; p = 0.0039 < 0.01); however, the released level of GLP2 in the rLV-GLP2-infected group was not significantly altered compared to the rLV-GLP2 plus pGFP-V-RS-c-Fos group (541.01 ± 84.28 versus 460.04 ± 124.85 pg/mL; p = 0.271 > 0.05) (Figure S7A). Furthermore, GLP2R was expressed in OB cells, and there was no significant difference among the rLV, rLV-GLP2, and rLV-GLP2 plus pGFP-V-RS-c-Fos groups (Figure S7B). As shown in Figure 8A, overexpression of GLP2 enhanced the expression of c-Fos, BMP, BALP, and PICP in OB cells compared to the rLV group. However, when c-Fos was knocked down, excessive GLP2 could not significantly alter the expression of BMP, BALP, and PICP in OB cells. Moreover, excessive GLP2 increased the luciferase activity of the promoter of BALP (Figure 8B), and it increased the activity of BALP in OB cells compared to control (Figure 8C). However, when c-Fos was knocked down, excessive GLP2 did not significantly alter the luciferase activity of the promoter of BALP and the activity of BALP in OB (Figures 8B and 8C). Furthermore, excessive GLP2 increased the positive rate of staining of BALP in OB (BALP-positive cells) compared to control (9.01% ± 1.55% versus 69.05% ± 11.6%; p = 0.0059 < 0.01). However, the c-Fos knockdown fully abrogated the function of GLP2 (9.01% ± 1.55% versus 10.89% ± 2.91%; p = 0.266 > 0.05) (Figures 8D and 8E).On the other hand, excessive GLP2 increased the luciferase activity of the promoter of PICP (Figure 8F) and increased the activity of BALP in OB compared to control (Figure 8G). However, when c-Fos was knocked down, excessive GLP2 did not significantly alter the luciferase activity of the promoter of PICP and the activity of PICP in OB (Figures 8F and 8G). Taken together, these observations suggest that the action of GLP2 is dependent on c-Fos in OBs.

**Figure 8:** c-Fos Knockdown Abrogates the GLP2 Action in the OB Cells (A) Western blotting with anti-GLP2, anti-c-Fos, anti-BMP,anti-BALP, anti-PICP in OB cells induced from MG63 infected with rLV, rLV-GLP2, rLV-GLP2 plus pGFP-V-RS-c-Fos. β-actin was used as an internal control. (B) The assay of luciferase activity of prmoter of BALP in OB cells induced from MG63 infected with rLV, rLV-GLP2, rLV-GLP2 plus pGFP-V-RS-c-Fos. **p < 0.01. (C) Cell BALP activity assay. Data are means of value from three independent experiments (error bar ± SEM; **p < 0.01). (D) The photography of BALP staining. (E) The BALP-positive rate in OB cells induced from MG63 infected with rLV, rLV-GLP2, rLV-GLP2 plus pGFP-V-RS-c-Fos. **p < 0.01. (F) The assay of luciferase activity of promoter of PICP in OB cells induced from MG63 infected with rLV, rLV-GLP2, rLV-GLP2 plus pGFP-V-RS-c-Fos. **p < 0.01. (G) Cell PICP activity assay. Data are means of value from three independent experiment (error bar ± SEM; **p < 0.01).

## Discussion

Recently, the role of GLP2 has been studied extensively, and a large number of studies have shown potential applications for GLP2 in disease therapy. In this report, we focused mainly on the view that GLP2 inhibits growth of osteosarcoma cells by inhibiting NF-κB and promotes direct differentiation of osteosarcoma cells to OBs dependent on c-Fos (Figure S8). To our knowledge, this is the first report demonstrating GLP2 is associated with osteosarcoma and OBs.

It is worth mentioning that our observations clearly demonstrated that GLP2 is crucial for the inhibition of osteosarcoma. Our results showed that GLP2 inhibits osteosarcoma cells growth elicited by NF-κB. This assertion is based on several observations: (1) GLP2 inhibits the expression and activity of inflammation-related gene NF-κB in osteosarcoma cells, and (2) excessive NF-κB fully abrogates the function of cancerous suppression of GLP2 in osteosarcoma cells. Our results imply that GLP2 is involved in the inhibition of development of osteosarcoma, which strongly suggests that GLP2 has suppressor properties. This is consistent with previous reports; for example, recent data have suggested the notion that GLP2 plays a key role in colon carcinogenesis.^21^

Furthermore, it is obvious that GLP2 promoted directed differentiation from osteosarcoma cells to OBs dependent on c-Fos. Herein, the involvement of GLP2 is supported by results from two parallel sets of experiments: (1) GLP2 increased the activity of BALP and PICP in OBs dependent on c-Fos, and (2) the depletion of c-Fos abrogated the GLP2 action in OBs. Our results imply that GLP2 is involved in the differentiation of osteosarcoma cells to OBs. This suggests that GLP2 may inhibit osteosarcoma progression by triggering differentiation of osteosarcoma.

Strikingly, our results showed that GLP2 inhibited the expression of c-myc, CyclinD1, and pyruvate kinase M2 (PKM2) dependent on NF-κB. It is well known PKM2 is a limiting glycolytic enzyme that catalyzes the final step in glycolysis, which is key in tumor metabolism and growth.^22^, ^23^ Moreover, PKM2 dephosphorylation by Cdc25A promotes the Warburg effect and tumorigenesis.^24^ In particular, PKM2 promotes tumor angiogenesis through NF-κB activation.^25^ Furthermore, cytosolic PKM2 stabilizes mutant EGFR protein expression through regulating HSP90-EGFR association.^26^ In particular, mutant EGFR is associated with tyrosine kinase, which plays a role in cancer.^27^ Moreover, it has been proven that c-myc and CyclinD1 play important roles during tumorigenesis.^28^, ^29^

Notably, our present observations also demonstrate that GLP2 decreased the interaction between β-catenin and NF-κB in osteosarcoma. β-catenin as intracellular signal transducer plays an important role in the WNT-signaling pathway. A report indicates that microRNA-153 promotes Wnt/β-catenin activation in hepatocellular carcinoma through the suppression of WWOX.^30^ Moreover, focal adhesion kinase (FAK) promotes OB progenitor cell proliferation and differentiation by enhancing Wnt signaling.^31^ A report also showed that long noncoding RNA BC032913 plays an inhibitory role in cancer aggression by inactivation of the Wnt/β-catenin pathway.^32^ In this report, our results suggest that GLP2 regulates and controls BMP. It is well known that BMP is critical for skeletal and cartilage development, homeostasis, and repair, which stimulate chondrogenesis of equine synovial membrane-derived progenitor cells.^33^ A study showed BMP-2 played a role in the differentiation of Runx2-deficient cells into OBs.^34^

In the report, we first proved that GLP2 exerts its effect in part through the upregulation of c-Fos and downregulation of NF-κB expression. Our present approaches provided unequivocal evidence for critical suppressor roles of the GLP2 in the tumorigenesis of osteosarcoma and osteogenesis, and they supported the notion that GLP2 may be an alternative bona fide inhibiting factor of osteosarcoma and promoting factor of osteogenesis. However, the exact mechanism underlying the role of GLP2 in the tumorigenesis of osteosarcoma and osteogenesis remains to be elucidated. We further explore the different pathways of GLP2 signaling to suggest suitable GLP2-based therapeutic strategies in cancer.

In conclusion, our results suggested that GLP2 promotes the osteogenic differentiation from osteosarcoma cells and inhibits the growth of osteosarcoma, indicating that GLP2 therapy could be a valuable approach to promote bone regeneration and to inhibit osteosarcogenesis. This may provide potential therapeutic targets for the treatment of osteosarcoma.

## Materials and Methods

### Cell Lines, Plasmid, and Lentivirus

Human osteosarcoma cell lines MG63 were obtained from the Cell Bank of Chinese Academy of Sciences (Shanghai, China). These cell lines were maintained in DMEM supplemented with 10% fetal bovine serum (Gibco BRL Life Technologies) in a humidified atmosphere of 5% CO_2_ incubator at 37°C. pGFP-V-RS and pGFP-V-RS-c-Fos were purchased from Origene (Rockville, MD, USA). pcDNA3 and pcDNA3-NF-κB were purchased from Addgene (Cambridge, MA, USA). rLV and rLV-GLP2 were purchased from Wu Han viraltherapy Technologies.

### Cell Infection, Transfection, and Stable Cell Lines

MG63 cells were infected with rLV and rLV-GLP2, respectively. MG63 cells were transfected with pGFP-V-RS-c-Fos and pcDNA3-NF-κB using transfast transfection reagent Lipofectamine 2000 (Invitrogen), according to the manufacturer’s instructions. We selected the single-cell clone with overexpressing GLP2 to establish the stable cell lines. Transfection efficiency was observed by Green imaging and measured by western blotting.

### Directed Differentiation of Osteosarcoma Cells to OBs

Direct differentiation of osteosarcoma cells were preformed by 0.1 μM dexamethasone(Dex), 0.5 mM β-glycerophosphate (β-GP) and 50 mg/L ascorbic acid (Asc) according to the manufacturer instruction. Alkaline phosphatase (ALP), Osteocalcin (Ocn), Bone morphogenetic protein (BMP), Procollagen I carboxyterminal propeptide (PICP) were detected in these cells according to the manufacturer instruction (TaKaLa).

### BALP Activity Assay

The BALP activity was adopted according to the manufacturer’s instructions (Beyotime). The sample, the detecting buffer, and para-nitrophenyl phosphate (p-NPP) were mixed and then incubated at 37°C for 5–10 min. Finally, 100 μL reaction stop solution was added to each well to stop the reaction, and then absorbance at 405 nm was measured.

### BALP Staining

The BALP staining was adopted according to the manufacturer’s instructions (COSMO BIO). The culture medium was removed and then each well was washed three times with 1 mL PBS. 500 μL 10% Neutral buffer solution was added to each, and the cells were fixed for 20 min at room temperature. Then, 10% Formalin Natural buffer solution was removed, and each well was washed with 2 mL deionized water three times. Then, 400 μL Chromogenic substrates was added to each well, and cells were incubated at 37°C for 20 min. Finally, cells were washed with deionized water to stop the reaction. The ImageJ software was used for the quantification of BALP.

### Alizarin Red S Staining

Cells were rinsed with 1× PBS 3 times and then fixed with formalin for 15 min. Following that, the cells were stained with alizarin red S for 5 min and then washed with PBS and dried and mounted.

### ELISA of GLP2

Diluted washing solution was filled into each hole of microplate and then the plate was shaken for 30 s. Then, the washing liquid was washed off and dried with absorbent paper (repeated 5 times). To each hole was first added the chromogenic agent A (50 μL) and then chromogenic agent B (50 μL). This was gently shaken to mix, avoiding light for 15 min at 37°C. Then, the microplate was taken out and termination liquid (50 μL) was added to each hole for reaction termination. The absorbance value (OD) of each hole was measured at 450-nm wavelength.

### RT-PCR

Total RNA was purified using Trizol (Invitrogen) according to the manufacturer’s instructions. cDNA was prepared by using oligonucleotide (dT)_18_ and a SuperScript First-Strand Synthesis System (Invitrogen). The PCR amplification kit (TaKaRa) was adopted according to the manufacturer’s instructions. PCR products were analyzed by 1.0% agarose gel electrophoresis and visualized by ethidium bromide staining using Image imaging system (Baygene).

### Western Blotting

The cells were lysed in RIRP lysis buffer and centrifuged at 12,000 × *g* for 20 min at 4°C after sonication on ice, and supernatants were separated. After being boiled for 10 min in the presence of 2-mercaptoethanol, samples were separated on a 10% SDS-PAGE and transferred onto nitrocellulose membranes, stained, and then blocked in 10% dry milk-PBS Tween-20 (TBST) for 1 hr at 37°C. Following three washes in TBST, the blots were incubated with antibody (appropriate dilution) overnight at 4°C. Following three washes, membranes were then incubated with secondary antibody for 60 min at 37°C. Signals were visualized by enhanced chemiluminescence (ECL).

### ChIP

Cells were cross-linked with 1% (v/v) formaldehyde for 10 min at room temperature and stopped with 125 mM glycine for 10 min. Crossed-linked cells were washed with PBS, resuspended in lysis buffer, and sonicated for 10 min in a SONICS to generate DNA fragments. Chromatin extracts were pre-cleared with Protein-A/G-Sepharose beads, and they were immunoprecipitated with specific antibody on Protein-A/G-Sepharose beads. After washing, elution, and de-cross-linking, the ChIP DNA was detected by PCR.

### RIP

Cells were lysed and the ribonucleoprotein particle-enriched lysates were incubated with protein A/G-plus agarose beads (Santa Cruz Biotechnology, CA) together with antibody or IgG for 4 hr at 4°C. Beads were subsequently washed and RNAs were then isolated for RT-PCR.

### Cell Proliferation Assay

Cells at a concentration 5 × 10^4^ were seeded into 96-well culture plates in 100 μL culture medium containing 10% fetal calf serum (FCS). Before detected, 10 μg/well cell proliferation reagent CCK8 (Yeasen) was added and incubated for 4 hr at 37°C and 5% CO_2_. Absorbance of OD450 was measured using SpectraMax M5 (Molecular Devices, MD, USA).

### Soft Agar Colony Formation Assay

5 × 10^2^ cells were plated on a 10-cm dish containing 0.5% (lower) and 0.35% (upper) double-layer soft agar. Then the 10-cm dish was incubated at 37°C in a humidified incubator for 14 days. Soft agar colonies on the 10-cm dish were stained with 5 mL 0.05% crystal violet for more than 1 hr and the colonies were counted.

### Transwell Assay

Transwell assays were performed in 24-well polyester (PET) inserts (Falcon 8.0-μm pore size) for migration assays according to the manufacturer’s instructions (BD Falcon). We observed and counted the migrated cells of triplicate membranes to determine the average migrated cell number.

### Xenograft Transplantation *In Vivo*

The 4-week-old male athymic BALB/c mice were injected at the armpit area subcutaneously with a suspension of 1 × 10^7^ MG63 cells in 100 μL PBS. The mice were observed 4 weeks and then sacrificed to recover the tumors. The wet weight of each tumor was determined for each mouse. The use of mice for this work was reviewed and approved by the institutional animal care and use committee in accordance with China NIH guidelines.

### Orthotopic Osteosarcoma Mouse Model

The model was carried out according to methodology as previously described.^35^, ^36^ Briefly, MG63 cells were cultured in DMEM and collected before transplantation, and they were resuspended in serum-free media to a final concentration of 10^7^ cells/mL. About 100 μL cell suspensions were injected into the right proximal tibia of 4-week-old female athymic BALB/c mice (a severe combined immunodeficiency mice). The mice were observed for 4 weeks and then sacrificed to recover the tumors. The wet weight of each tumor was determined for each mouse. The use of mice for this work was reviewed and approved by the institutional animal care and use committee in accordance with China NIH guidelines.

### Statistical Analysis

Each value was presented as mean ± SEM, with a minimum of three replicates. The results were evaluated by statistical software (SPSS), and Student’s t test was used for comparisons, with p < 0.05 considered significant.

## Author Contributions

Study & Experimental Design, Y.H.; Experimental Operation & Data Analysis, Y.L. and D.L.; Manuscript Preparation, Y.H. and Y.L.; Manuscript Review & Editing, Y.H.; Funding Acquisition, Y.H.

## Conflicts of Interest

The authors disclose no conflicts of interest.

## Supplemental Information

Document S1. Figures S1–S8

Document S2. Article plus Supplemental Information
